# Non-invasive Prenatal Testing, What Patients Do Not Learn, May Be Due to Lack of Specialist Genetic Training by Gynecologists and Obstetricians?

**DOI:** 10.3389/fgene.2021.682980

**Published:** 2021-06-17

**Authors:** Thomas Liehr

**Affiliations:** Institute of Human Genetics, Jena University Hospital, Friedrich Schiller University Jena, Jena, Germany

**Keywords:** non-invasive prenatal testing, qualified genetic counseling, cell-free placental DNA, massively parallel sequencing, single nucleotide polymorphism whole genomic sequencing, background knowledge, NIPT-short-cuts

## Abstract

Platforms for “non-invasive prenatal testing” (NIPT), or also referred to as “non-invasive prenatal screening” (NIPS) have been available for over 10 years, and are the most recent tools available to obtain information about genetic condition(s) of an unborn child. The highly praised advantage of NIPT-screening is that results can provide early hints on the detection of fetal trisomies and gonosomal numerical aberrations as early as the 10th week of gestation onward, without any need for invasive procedures, such as amniocenteses or alternatives. Understandably, the public along with gynecologists and obstetricians eagerly await these early test results. Their general hope for normal (=negative) test results is also justified, as in >95% of the tested cases such an outcome is to be expected. However, pregnant women can be disappointed and confused, particularly regarding the genetic information and proposed care when the results are positive, and these emotions are also common with false-positive and false-negative NIPT results. Finally, such concerns in understanding the advantages and limitations of this routinely ordered screening tool end up at Clinical Geneticists and Genetic counselors. In this review, general background on NIPT, differences of NIPT platforms, advantages and limitations of NIPT, as well as consequences of insufficient counseling before and after NIPT are summarized. To provide comprehensive care in all pregnancies situations, professionals need a careful attitude toward offering NIPT along with specially training and qualifications in counseling for these procedures. Often it is gynecologists and obstetricians who discuss the use of NIPT with patients; however, although these physicians have a highly qualified background and knowledge in their respective specialty area(s), they may lack specific training on the interpretation of NIPT-screening results. These potential knowledge gaps must be closed quickly and comprehensively by the corresponding scientific societies to ensure optimal patient care.

## Introduction

Advances in modern medicine are in parts breathtaking when compared to our limited capabilities only 2, 5, or 10 decades ago. This is especially true for prenatal predictive genetic testing in human reproduction. Today it is hard to imagine reproductive care without many of the tools and approaches now available, which enhance the study and evaluation of the life of the unborn. These enumerable invasive and non-invasive approaches allow examination of the fetus and may detect genetic condition(s) (Hixson et al., 2015). All these evaluation possibilities are, from the pregnant mother’s perspective, just options she must choose from to answer the single burning question: “How likely is it that this baby in my womb will be affected or not affected by a (specific) genetic disease?” Or more simply: “Will my baby be okay?” With respect to the desire for negative results and for those who may use these results to decide on an induced abortion in the presence of a fetal anomaly, the pressing need for early test-results is completely understandable (Hixson et al., 2015; Liehr et al., 2017).

Pregnant women seek help, education, and counseling regarding these tests primarily from their gynecologists and obstetricians. Also many national health system regulations require qualified genetic counseling before and after NIPT either from gynecologists or obstetricians, and/or genetic counselor or a medical doctor (MD) with a specialization in Clinical Genetics (which may but must not include gynecologists or obstetricians) (Skirton, 2018). During qualified genetic counseling, a general risk-estimation is performed first for the pregnancy and can simply base on epidemiological data, including family history of disease(s) and/or abortion(s), age, ethnicity, and weight of pregnant woman. Suitable testing options can then be discussed and ideally, after counseling and time for consideration of available options, the pregnant woman/the couple should be allowed to form their own educated decision on the need for further genetic tests, and if so, which one(s) she/they want to undertake for the evaluation of the fetus (National Society of Genetic Counselors’ Definition Task Force et al., 2006).

In many countries ultrasonography is part of routine prenatal testing and is offered free of charge for all pregnancies (Hixson et al., 2015). It remains the most straightforward non-invasive method to learn about the condition of an unborn child—test accuracy is estimated at up to 82% (Levi, 2002). First trimester sonography is an important and integral part of comprehensive first trimester screening (FTS) (Anderson and Ghaffarian, 2021). FTS also includes additional biochemical testing of maternal blood for pregnancy-associated plasma protein A (PAPP-A) and free β-human chorionic gonadotropin (β-hCG) (Rink and Norton, 2016), which also take into account maternal age, ethnicity, and body weight. Using FTS, a 91–96% reliable risk estimation for the fetus can be achieved (Hixson et al., 2015). However, if an enhanced risk has been identified, further clarification and/or testing may be required to determine if the underlying problem is one of the more common trisomies of 13, 18, or 21, or any other “genetic problem,” or to confirm a false positive finding. Therefore, until recently, the only options available after abnormal sonography were invasive prenatal diagnostic approaches—i.e., amniocentesis (AC), chorionic villi (CVS), and/or umbilical cord blood sampling (CBS), which differ in the tissue examined; in CVS the placenta is studied, whereas in AC and CBS real fetal tissues are examined. Overall, discussions of the procedure and result expectations regarding all aforementioned prenatal testing approaches, which have been available for more than two decades, are well understood by patients and medical doctors (Hixson et al., 2015; Liehr et al., 2017).

However, in the last decade, another, new approach has become routinely available and has subsequently joined the plethora of other prenatal testing approaches—the so called “non-invasive prenatal testing” (NIPT) or also “non-invasive prenatal screening” (NIPS) (Skrzypek and Hui, 2017). This recent development in prenatal diagnostics is based on the so-termed second-generation sequencing approaches for analyzing copy number alterations in free placental DNA in maternal blood plasma (also referenced in the literature as cell-free fetal DNA = cffDNA; see also below) (Liehr et al., 2017). NIPT is advantageous given DNA derived from the placenta (!) during pregnancy can be examined very early (at around 10th week of gestation = w.o.g.) for the most frequent chromosomal aberrations detected in the first and second trimester (Taylor-Phillips et al., 2016). With the widespread utilization of NIPT screening, more and more countries have added the assay as a statutory health insurance benefit, however, in tandem, moral concerns regarding the use of the tests in pregnancy decision making have been raised, e.g., concerns over the use of the results in decision making for or against continuing a current pregnancy (Farrell et al., 2014). In addition, Nigün Dutar (Institute for Prenatal Medicine and Ultrasound, Wuppertal, Germany) recently stated: “The diagnostic gain of the non-invasive prenatal tests is actually very small. On the other hand, the pressure on pregnant women to give birth to a perfect child will increase due to a blood test that is supposedly easy to use” (translated from German site: https://www.aerzteblatt.de/nachrichten/99669/Praenatalmediziner-warnen-vor-breitangelegtem-Einsatz-nichtinvasiver-praenataler-Tests). However, in disagreement with the public suggestion that NIPT may be “a blood test that supposedly easy to use,” there are several points as outlined below that must be brought to the attention of the field.

## NIPT Is Not Equal to NIPT

NIPT was developed based on the 1997 finding that in the blood, or more accurately in plasma of a pregnant woman, there is cell free **placenta**-derived DNA along with maternal cell-free DNA (Lo et al., 1997). This DNA derived from the placental syncytiotrophoblast layer is misleadingly referred to as cell-free **fetal** DNA (cffDNA) in literature (Shaw et al., 2020). This free placenta-derived DNA can be detected earliest at ∼4.5 w.o.g. (D’Aversa et al., 2018) and can reach 30% of cell-free DNA in a pregnant woman during the 3rd trimester. Following birth, placental cell-free DNA is removed from maternal blood within hours, and as such, no mix-up of genetic materials from different pregnancies is possible (Lo et al., 1999; Shaw et al., 2020).

In the NIPT-literature, it is often difficult to understand which NIPT protocol, method or evaluation platform was used by the authors, and which genetic aberrations were potentially detectable by a specific test. Generally, it is less cumbersome when commercial NIPT assays are performed because in most cases these vendors declare the use of a second generation sequencing based testing approach and they provide results as Z-scores, with normally high positive predictive values (PPVs) and with detailed sensitivity and specificity of the test:

- A Z-score of more than 3 standard deviations away from the expected value for the DNA fragments derived from a specific chromosome is considered a high-risk-result for trisomy (Palomaki et al., 2011).
- The sensitivity of NIPT for trisomy 21 is generally given as 99.3%, for trisomy 18, 97.4% and for trisomy 13, 97.4%,
- with a specificity of 99.9% for trisomy 21 (Taylor-Phillips et al., 2016).
- Previous PPVs for trisomy 21 were given as 80–90% however, they are now corrected to 45.5% and lower (Skrzypek and Hui, 2017).

Thus, these “standard NIPT” protocols are able to detect trisomies 13, 18, and 21 and gonosomal numerical aberrations. When further copy number alterations are detectable by a NIPT platform, such as trisomies of other chromosomes, or specific microdeletion and microduplication syndromes (MDDs) (Weise et al., 2012), these protocols are marketed as “expanded NIPT” or “NIPT Plus” tests. For these emerging platforms, the data for Z-scores, sensitivity, specificity and PPVs are in most cases hard to find or are not provided (Skrzypek and Hui, 2017; Shaw et al., 2020; Ye et al., 2021).

The following whole genomic sequencing (WGS) based principles are used to perform a NIPT:

(i) shotgun massively parallel sequencing (s-MPS),
(ii) target massively parallel sequencing (t-MPS) and
(iii) single nucleotide polymorphism (SNP) based WGS.

In both MPS based approaches either untargeted (s-MPS) or targeted (t-MPS) regions of the pregnant mother’s cell-free DNA are sequenced. An aneuploidy is indicated as an excess (or deficit) in the detected amount of DNA for the studied chromosome compared with the expected result for diploid cases. In this evaluation, maternal and placental DNA cannot be distinguished, and only s-MPS based NIPT tests can be widened to become “expanded NIPT” or “NIPT Plus” tests. In SNP-based NIPT, maternal and placental DNA can be distinguished, and thus the relative contribution of both DNA-types is measured; with this approach “expanded NIPT” can be easily performed (Neveling et al., 2016; Skrzypek and Hui, 2017; Andari et al., 2020). In addition, slightly alternative approaches have been reported, such as the use of real-time polymerase chain reaction before low coverage DNA sequencing (Chen et al., 2013). All current WGS platforms are considered to be suitable for NIPT (Neveling et al., 2016).

Thus, it must be stated that all commercial NIPT tests and all published NIPT data should be analyzed in detail to confirm the underlying approach used for the assay. Optimally, data should be available for sensitivity, specificity and PPVs, as well as cut-off levels, which should include the number of false negative and false positive results to be expected for the corresponding NIPT approach. However, this data is often not readily available, sometimes even impossible to obtain, as in many cases the approaches are patented and quite often, the approach used to obtain and calculate results remains a coveted company secret. Accordingly, it is also difficult to align different publications for NIPT-screening and a paucity of literature is available for such comparisons (Agarwal et al., 2013; Kotsopoulou et al., 2015; Sekelska et al., 2019). While most companies started with NIPTs to offer testing for trisomy 13, 18, and 21 as well as gonosomal aberrations, more and more offer and are now testing for additional genetic conditions (with the anticipated added expense) (Liehr, 2019), and a few platforms also test all chromosomes, but fail to appropriately identify which MDDs were under evaluation by the platform (Health Quality Ontario, 2019).

Even more complexity in testing within the field is exemplified by differences in testing, e.g., Belgium and the Netherlands have offered NIPT since 2017 to all citizens, which are whole genome oriented assays that also include evaluation of genetic material associated with certain monogenic disorders (van Schendel et al., 2017; Žilina et al., 2019). Further evidence of confusion within the field comes from the naming convention used for the first NIPT (also called NIPS) assays, in contrast to testing for single-gene disorders on free placental DNA, referred to as “non-invasive prenatal diagnosis” (NIPD). Thus, as Shaw and colleagues provocatively wrote in 2020: “The distinction between diagnostics and screening has become blurred, and there is a clear need for the education of physicians and patients regarding the technical capabilities and limitations of these different forms of testing. Furthermore, there is a requirement for consistent guidelines that apply across health sectors, both public and commercial, to ensure that tests are validated and robust and that careful and appropriate pre-test and post-test counseling is provided **by professionals who understand the tests offered**.” This statement is further supported by the statement of Stefanovic (2019): “**The knowledge and counseling should be substantially improved**. Cell-free DNA screening is not a replacement for diagnostic testing and its use in prenatal testing is complex and limited” (Stefanovic, 2019).

## NIPT: Advantages and Short-Cuts

NIPT is advantageous given DNA derived from placenta during pregnancy can be tested for the most frequent chromosomal aberrations generally detected in the first and second trimester; this can be performed starting around the 10th w.o.g., with a result anticipated within 2 weeks. Thus, information on the health of an unborn child can now be obtained a few weeks earlier than by FTS or invasive approaches. Accordingly, expecting couples have long awaited this new possibility and in only a few years, NIPT has rapidly transformed prenatal care worldwide. Thus, massive reduction in the number of invasive prenatal procedures performed has already been observed (Shaw et al., 2020). Even with these reported changes in care pathways, surprisingly, the aforementioned is the only relevant summary of all publications regarding the appropriate advantages of NIPT. The following list of potential problems is much longer, and unfortunately, these issues are not as well-known to the public and/or gynecologists and obstetricians when compared with the widespread awareness of the catchy statements often used in favor of the technique (see also Table 1).

**TABLE 1:** Expectations and reality of NIPT.

NIPT	
Expectations	Reality
The test can be performed earlier than others	This is correct; it is a screening test
The test includes zero risk for the unborn baby in contrast to invasive testing, which has 1–3% abortion risk	First point is correct; however, nowadays risk of invasive testing is between 0 and 0.3% only
If we do the NIPT there is no need to do invasive testing	In case NIPT is positive an invasive confirmatory test is obligatory In case NIPT is negative but sonography normal invasive confirmatory test is recommended to exclude a placenta mosaicism
The test is based on fetal DNA	The test is based on placenta derived DNA
The test is a quick test and is easy to understand	There are many variants of the test There is a need for detailed pre-test counseling (e.g., to explain that a hidden maternal tumor may be detected) The technical details how the test works are very complicated
The test is equally reliable for all kinds of genetic conditions tested	Highest reliability is available for trisomy 21; all other conditions have lower PPVs In many cases there are no PPVs available for the corresponding tested syndrome
There is a clear answer if baby will be ok.	It is a screening test
The results are available very fast	It lasts ∼2 weeks and in 1.58–6.39% of the cases the tests needs to be repeated due to not sufficient cffDNA in maternal plasma
There is a clear answer if baby will be not ok, e.g., have trisomy 21	2% risk of placenta mosaics; false positive results are possible
It is a test which can exclude all genetic problems	Neither the “normal NIPT” nor the “expanded NIPT” can exclude all possible genetic conditions

The list of limitations begins with the understanding that is important to keep in mind: “NIPT is a screening test, with positive results requiring confirmation via invasive testing” (Shaw et al., 2020). In addition, negative NIPT results and a fetus with sonographic findings may need further (invasive) testing (Liehr et al., 2017). As long as no (really reliable) “expanded NIPT” or “NIPT Plus” test is available it must be understood and considered that at a maximum 50% of cases with chromosomal aberrations of the first and second trimester are detectable via NIPT. Accordingly, as reported in 2016, the extensive use of NIPT in United States since 2011 has been associated with a dramatical increase in the rate of newborns with MDDs as compared with previous years (Beaudet, 2016).

Furthermore, the misleading use of the name cffDNA instead of free placental DNA has further implications on the general understanding of this assay. It is known, and confirmed by many “single case reports” in the literature, that genetic and chromosomal conditions of placenta are different from that of the fetus in 2% of cases (in second trimester) and may be even higher in first trimester evaluations (Hartwig et al., 2017). Thus, a negative NIPT can only exclude ∼98% of adverse copy number changes in the fetus, and a positive NIPT for a trisomy can be false positive in up to ∼2% of the cases. The phenomenon of confined placental mosaicism is real, and should be understood when interpreting the NIPT-screening findings or while providing pre/post-test counseling (Lau et al., 2014; Hartwig et al., 2017; Liehr et al., 2017).

In the beginning of NIPT-era, which continues today by some vendors, NIPT is advertised as an assay capable of reducing the risk for invasive tests. This erroneous claim ignores two facts: (i) that invasive testing is still necessary in the case of a positive NIPT; and (ii) that the terrifying data often touted of 1–3% abortion risk associated with CVS, AC or CBS is derived from outdated studies performed in the 1980s/1990s. That is, these data are derived from a time that predated the availability of better suited needles for aspiration and the routine control of the procedure by sonography. Today, the risk of invasive diagnostics is at 0–0.3% (Liehr et al., 2017). This is an important distinction regarding invasive procedural risk, which is critical data pregnant women must be properly informed about when considering available testing options during pregnancy.

False positive results can also derive from maternal (acquired) mosaicism in peripheral blood or come from other tissues excreting cells and cell-free DNA into the plasma of the pregnant woman. Cases have been reported where a previously undetected maternal malignancy was the reason for an abnormal NIPT result (Bianchi et al., 2015; Saes et al., 2019). Other abnormal NIPT outcomes have been reported to result from maternal mosaicism (mos 46,XX/45,X), leading to incorrect conclusions regarding a sex chromosome abnormality in the fetus (Wang et al., 2014). Furthermore, other studies report that MDDs in the mother have been falsely attributed to fetus (Kumps et al., 2020). Lastly, a chromosomally abnormal vanishing twin can also interfere with the NIPT-result; in particular, targeted SNP-sequencing based NIPT cannot distinguish between triploidy and vanishing twin scenarios (Andari et al., 2020).

Finally, it also possible, as observed in 1.58–6.39% of NIPT-tests, that free DNA in the pregnant mother’s blood does not contain sufficient placental DNA to achieve an informative test result. This issue is of great concern when performing NIPT-screening in early w.o.g. and/or if mother is obese, because in these situations, the ratio of placental/maternal cell-free DNA is altered, leading to a disadvantage when attempting to detect placental derived DNA (Skrzypek and Hui, 2017). Interestingly, failure rates differ according to the NIPT-technology: NIPT based on MPS have the lowest and targeted SNP-sequencing have highest failure rates (Yaron, 2016).

All the points raised herein must be discussed in a qualified genetic counseling before NIPT is consented and performed. This level of understanding of both the capabilities and limitations of NIPT-screening is only possible if gynecologists and obstetricians either provide this appropriate counseling or refer the pregnant woman/the couple to a counselor or MD with specialization in Clinical Genetics (Skirton, 2018). Logically, such counseling requires considerable care and time, which may be not readily available in routine daily practice of the doctor’s office.

## Consequences of Insufficient Counseling Before and After NIPT

The most obvious and worst possible outcome imaginable from a lack of sufficient counseling are that the families consented for NIPT do not understand the implications of the test performed (Table 1). The following three examples support the need for appropriate counseling:

- Beaudet (2016) reported an increase of newborns with MDDs after massive introduction of NIPT in United States. This is most logically due to a misunderstanding by pregnant women that a negative NIPT means the baby will be genetically normal, and that all possible genetic aberrations have been “ruled out” by this test, even when there were hints of malformations observed in FTS or sonography.
- In the same vain, are many cases repeatedly observed by the author of this paper: when using MPS-based NIPT it is possible to detect trisomies, but not triploidies. This fact is difficult for laymen to comprehend and in some cases following a normal NIPT, the pregnant women learned of the triploid condition only after an AC. This is likely due to a failure in consultation to explain the limitations of the test, which may lead to a break down psychologically, as without all of the information they were inappropriately convinced up to this moment that the normal NIPT result all but assured them they will deliver a healthy child.
- Similarly catastrophic are prenatal cases that are voluntarily terminated after an abnormal NIPT screening, without any verification by sonography and/or invasive procedures of a false positive finding, which are also reported in literature (Xue et al., 2020).

NIPT is commercialized and advertised as an assay that will provide early information on the unborn child that is quick and with clear answers, which will most often provide the optimal and hopeful anticipated result desired by the pregnant mother: no genetic abnormalities are found. But how well can gynecologists and obstetricians answer questions in cases of a delayed or abnormal result? Here is an example based on the experience of one of ∼25 women, the author was in contact with, and who was interviewed by a German newspaper (Krafft, 2020):

- The woman got a NIPT result that her baby could have a trisomy 18. She did not feel well-informed after getting the result from her obstetrician and was not referred to a genetic counselor to discuss the findings. After AC and nearly ∼8 weeks after the NIPT she received information the baby was okay—the abnormal result was most likely associated with confined placental mosaicism. Her comment to the journalist was “I was psychologically exhausted. For weeks. In retrospect, I think to myself that I should never have taken this test” (translated from Krafft, 2020).

Further examples, known to the author of this paper include situations where pregnant women were desperate for clarity following an abnormal NIPT test; many of them had already received further results after invasive diagnostics and Clinical Genetic counseling, which was in the majority not referred appropriately by their gynecologists and obstetricians; instead they found a suited counselor after performing their own internet research. Problems associated with NIPT-screening results these women did not get a qualified answer from gynecologists and obstetricians are as follows:

- What is a chromosomal mosaic and a supernumerary marker chromosome?
- The pregnant women were told in such cases that a special trisomy was indicated by NIPT, but afterward in AC there was only a hint on a mosaic trisomy and/or a small supernumerary marker chromosome (sSMC) (Liehr, 2021). In such cases genetic specialists need to explain that a mosaic can possibly reduce the expected abnormal phenotype, that an sSMC is in ∼70% of cases a kind of harmless leftover from a trisomic rescue. Yet the author knows five such cases who were in direct contact with him.
- Why is the accuracy and PPV of the test only 5% in my case?
- This question was asked by a pregnant woman, who received the result of a “extended NIPT” with the information—all is okay, but there is a 5% risk for a specific MDD—which could have been 1p36. A molecular cytogenetic test on AC derived cells excluded a corresponding microdeletion and subsequently a healthy child was born. This example highlights the limitations of many extended NIPT platforms, i.e., these companies do not have reliable cutoff rates, and the reporting is somewhat ambiguous, often leading to uncertainty in the results, which is also difficult to reconcile for the patient following a short consultation with a gynecologist or obstetrician, who may also be puzzled by such a test outcome.

## Concluding Remarks

As discussed herein, all of the aforementioned issues are of high ethical impact for societies worldwide. However, a more careful approach for offering NIPT along with a new way of counseling have recently been suggested, which may serve to enhance patient care (Kater-Kuipers et al., 2020). Education and training must ensure that gynecologists and obstetricians can perform their role as the primary provider of NIPT advisement though awareness of all implications for the pregnancy that may be associated with the test results. Concrete normative measures for application of NIPT have already been published (Guidelines of the Royal College of Obstetricians Gynecologists, 2019; American College of Obstetricians and Gynecologists’ Committee on Practice Bulletins—Obstetrics, Committee on Genetics, Society for Maternal-Fetal Medicine, 2020); still normative measures for educational level of MDs need to be established by the corresponding national societies. In most countries ongoing education is anyway obligatory for MDs. Thus, corresponding courses providing details on NIPT-testing, -advantages and -limitations should be offered by national medical societies, held by independent laboratory specialists rather than company representatives. Connected with this could be a certificate allowing for offering NIPT only if an MD has this kind of advanced training.

Overall, information from this review, from commercial NIPT providers, and many recent NIPT publications provide evidence that alternative and more reliable approaches such as FTS may be underestimated, and that limitations and issues of NIPT must be widely distributed by appropriate professional societies.

## Author Contributions

The author confirms being the sole contributor of this work and has approved it for publication.

## Conflict of Interest

The author declares that the research was conducted in the absence of any commercial or financial relationships that could be construed as a potential conflict of interest.
